# Modeling Adoption Behavior of Prefabricated Building with Multiagent Interaction: System Dynamics Analysis Based on Data of Jiangsu Province

**DOI:** 10.1155/2021/3652706

**Published:** 2021-11-30

**Authors:** Zhen Li, Shaowen Zhang, Qingfeng Meng

**Affiliations:** School of Management, Jiangsu University, Zhenjiang 212013, China

## Abstract

In recent years, the development of prefabricated building (PB) mode in China has gradually attracted the attention of stakeholders. It is of great significance to explore the adoption behavior of PB mode by Chinese construction enterprises. Using the method of combining evolutionary game theory with system dynamics and considering the multiagent interaction of the government, construction enterprises, and consumers, as well as the influence of multiple factors, this paper constructs a model of construction enterprises' adoption behavior of PB mode. The purpose is to clarify the mechanism of Chinese construction enterprises' adoption behavior of PB mode and the evolution law of market share. The research results show the following. Firstly, government subsidy plays an important role in promoting the maturity of PB market, but it plays a relatively small role in the more mature and stable market. Secondly, the higher the initial acceptance probability of the construction enterprise, the greater the peak of the PB market share and the greater the volatility, but it has no differential impact on the balance of the PB market in the later stage. Thirdly, price factors and quality factors, respectively, have an important impact on the increase of the PB market share in the early and late stages of the formation of the PB market, but the delivery waiting time factor has no significant impact on the PB market share.

## 1. Introduction

The construction industry occupies a pivotal position in the national economy of all countries in the world, but it is also one of the industries with a high degree of energy intensiveness [1, 2]. It has always had problems such as high carbon emission and serious energy consumption. For example, the annual carbon dioxide generated by global construction accounts for more than 40% of the world's total carbon dioxide emission, and the annual energy consumed accounts for more than 30% of the world's total energy consumption [3–5].

The traditional construction mode has the problems of high pollution and high energy consumption during the construction period, which is not in line with the modern development concepts such as energy conservation and emission reduction and green and sustainable development [6]. In order to promote the green and sustainable development of the construction industry, the prefabricated building (PB) mode has been gradually introduced into China. PB mode not only has the advantages of improving production efficiency, reducing construction cost, and increasing construction safety but also has the functions of reducing carbon emission, reducing energy consumption, and reducing construction waste [7, 8]. Therefore, the Chinese government pays more and more attention to the transformation from traditional construction mode to PB mode and tries to promote the development of PB by means of encouraging technological innovation and policy incentives such as subsidies [5]. The Chinese government stipulates that by 2020, 15% of new buildings nationwide (according to the floor area) will be constructed using the PB mode each year, and this proportion will increase to 30% by 2025 [9]. However, the current application and promotion of the PB mode is not ideal.

In fact, the application and promotion of PB mode in China faces many obstacles. For example, in terms of the government, there is a lack of detailed government policy formulation and effective incentives [10]. In terms of the industry, there is a lack of specific construction specifications and construction standards for prefabricated buildings [11]. In terms of market demand, there are obstacles such as insufficient consumer awareness of PB and insufficient market demand [12, 13]. Therefore, considering the significance of promoting PB mode in China and many obstacles it faces in the development process, it is necessary to model and analyze the adoption behavior of the PB mode by construction enterprises in the context of multiagent interaction.

Modeling and analyzing the behavior of construction enterprises adopting PB mode and then understanding the mechanism of the adoption of PB mode play an inestimable role in the development of the whole industry. Some scholars have conducted relevant research on the factors affecting the adoption and promotion of the PB mode. For example, Li et al. [14] believe that the prefabricated component subsidies implemented by the government have a positive impact on the use of prefabricated components and the improvement of construction performance. Multiple policy measures are mutually complementary, and the combined effect of these policy measures is greater than the sum of the effects of individual policy measures. Wei et al. [15] believe that the promotion of government policies and the leadership of construction enterprises are the main driving factors to promote the development of PB. Research by Gan et al. [7] showed that strengthening policies and regulations has a strong stimulating effect on the promotion of PB and has a significant effect on solving organizational and environmental problems in the promotion process, but the effect on solving technical problems is not ideal. However, Xiahou et al. [16] found that in order to promote PB mode, China needs not only the promotion of the government and the pull of the market environment but also the self-driving of the PB industry. It is pointed out that the main way to promote the development of China's PB is to transform and upgrade the traditional construction industry and solve the development difficulties.

Some scholars believe that the government plays an important role in the process of whether the PB mode is adopted by the construction enterprise [5]. Government policy incentives have a positive effect on the promotion of PB mode, and reasonable policy incentives can help reduce opportunistic behavior [17, 18]. However, policy documents tend to favor the environment and supply and lack policy measures for other areas [7]. Currently, government subsidies are the main way to promote the development of PB mode, but in the long run, continuous government subsidies are not a long-term solution to maintain the steady development of the industry. At the same time, the government's publicity and guidance work is also gradually starting. For example, Xi'an, China, has begun to encourage consumers to purchase prefabricated commercial residential buildings and promote the development of prefabricated buildings from the consumer level.

Secondly, the construction enterprise is also one of the most influential stakeholders in the PB industry [19]. As the investor of a construction project, the construction enterprise's behavioral willingness and adoption behavior are highly correlated [20]. Therefore, whether the construction enterprise adopts the behavior and decision making of PB mode is very important for the development of the PB industry. The construction enterprise will make reasonable decisions on its own construction mode based on the economic benefits, environmental performance, maintenance cost, and other factors of the construction project [21, 22]. However, the high initial cost of adopting PB mode is one of the main factors that hinder the construction enterprise from adopting PB mode [7, 23]. The poor overall efficiency of PB industry also leads to the lack of motivation for some construction enterprises to adopt PB mode [13].

In addition, whether the PB mode is adopted is closely related to market demand [24]. The purchase motivation of consumers will have an important impact on the development of the PB market. Due to the lack of Chinese consumers' understanding of PB [12], Lee and Kim [25] believe that it is necessary to increase the correct publicity and guidance to change consumers' attitudes towards PB. Some scholars have studied consumers' attention to PB and the evolution trend of their attention content. For example, Wang et al. [26] pointed out that although consumers' attention to PB fluctuates greatly, it shows an overall upward trend, and the introduction of relevant government policies will significantly affect consumers' attention. Hu et al. [27] found that the content of PB that consumers are most concerned about mainly involves high-quality building performance.

In summary, the behavior and decision making of the construction enterprise adopting the PB mode are affected by multiple stakeholders. Existing research studies have identified the stakeholders who influence the adoption of the PB mode and analyzed the influencing factors and their effects. However, it rarely involves the influence of consumer group decision making on the adoption of the PB mode. In addition, less consideration is given to the complex interaction between a large number of factors and their nonlinear effects on the adoption behavior of PB mode.

In fact, first of all, consumers' cognition of PB and purchasing decisions are of great significance to the adoption of the PB mode. Consumers' purchase decision making is a more complex process, which considers many factors, such as price, quality, delivery waiting time, and so on. Previous studies generally regarded consumer demand as an exogenous variable to analyze its linear relationship with the adoption behavior of PB mode. This paper constructs a more realistic consumer decision-making model, which plays a vital role in revealing deeply the adoption behavior of PB and the evolution of market competition in the context of multiagent interaction. Secondly, the adoption behavior of PB mode by construction enterprises is also affected by many subjects and factors. They will comprehensively consider government policies, the status quo of the industry, market demand, and competitive pressure and adopt a suitable construction mode in the pursuit of maximizing their own economic benefits. Therefore, there are relatively complex dynamic interactions between construction enterprises and between construction enterprises, government, and consumers. In the process of studying the adoption behavior and mechanism of PB mode, this dynamic and complex interaction and game relationship cannot be ignored [9].

To sum up, on the basis of considering more realistic consumer purchase decisions and more complex interaction among multiple subjects, this paper will focus on the analysis of the adoption behavior and mechanism of the construction enterprise to PB mode under the scenarios of government subsidies to the construction enterprise, government publicity and guidance to the market, PB products with different prices, qualities, and delivery waiting times, and different adoption intentions of the construction enterprise. This paper attempts to provide a theoretical basis for improving the market competitiveness of PB products and formulating reasonable policies and measures for the government. This is of great significance for the Chinese construction industry to achieve energy saving and emission reduction targets and to practice the concept of green and sustainable development.

This research considers the complex interactions among stakeholders (government, construction enterprises, and consumers) that influence the adoption of PB mode and the bounded rational behavior of decision-making. This research also considers many obstacles in the process of adopting PB mode, as well as the complex interaction and nonlinear feedback relationship between these factors. This research will use the method of system dynamics to model and analyze related problems. System dynamics are more suitable for analyzing complex systems. This method can be used to understand the behavior of the system over time and the relationship between the system structure and decision rules [28]. Also, in the process of Chinese construction enterprises adopting PB mode, the bounded rational game between them and industry competitors is continuous. Therefore, the behavior of both parties must be discussed from a dynamic perspective [9]. Evolutionary game theory has been widely used in the study of bounded rational behavior, such as the study of stakeholders in the construction industry [29]. Therefore, this paper will use the research method of combining evolutionary game and system dynamics to model and analyze the behavior and mechanism of PB mode adopted by construction enterprises in China. It hopes to provide a theoretical basis for the rapid and sustainable development of PB mode in China.

This paper attempts to solve the following three problems:

1. What impact will government subsidies and government propaganda and guidance have on the adoption behavior of PB mode by construction enterprises?
2. What impact will the initial willingness of Chinese construction enterprises to adopt PB mode have on the diffusion and evolution of the follow-up market of PB mode?
3. What kind of evolutionary trend will the market proliferation of PB products under different prices, qualities, and delivery waiting times be?

## 2. Model

This paper combines evolutionary game theory with system dynamics to model and analyze the relationship and behavior of the three subjects involved in the adoption of PB mode: government, construction enterprises, and consumers.

### 2.1. Evolutionary Game Model

The construction enterprise will make decisions on the specific construction mode of the project. One is the adoption of traditional cast in situ buildings (TB) (hereinafter referred to as “*D*_*N*_”). The second is the adoption of PB (hereinafter referred to as “*D*_*Y*_”), including the selection of qualified and capable design institutions for modular design of drawings, the production of prefabricated components by prefabricated component manufacturers, and the assembly construction by construction organizations.

Whether the construction enterprise adopts PB mode will be mainly affected by government subsidies, competition from the same industry, consumer demand, and other factors. The interaction relationship and decision-making mechanism between agents are shown in Figure 1.

In order to clarify the competition mechanism among construction enterprises and then construct a system dynamics model with multiagent and multifactor comprehensive influence, this paper first uses the evolutionary game method to construct the behavior rules for construction enterprises to adopt PB mode. The construction enterprises are divided into two groups: initial adoption (Type Y construction enterprises) and initial nonadoption (Type N construction enterprises) of PB mode.

In the given situation, the two groups will take different strategies to play the game. This paper makes the following assumptions for model construction:

Hypothesis 1: assume that the overall number of construction enterprises remains unchanged. The construction enterprise will select a strategy that suits itself based on certain rules in each time unit.
 Hypothesis 2: “*D*_*Y*_” will increase the construction cost of the project. Use *x*_*Y*_ to represent the probability of the “*D*_*Y*_” strategy and *x*_*N*_ to represent the probability of the “*D*_N_” strategy, where *x*_*N*_=1 − *x*_*Y*_, and *x*_*Y*_ and *x*_*N*_ are all functions of time *t*.
 Hypothesis 3: the construction enterprise will choose its strategy according to its own profit level. The construction enterprise will compare its payoff with that of its competitors, so as to choose a strategy to make its expected payoff higher. Type Y construction enterprises and Type N construction enterprises will calculate their respective payoff differences. Taking Type Y construction enterprises as an example, if their payoff difference is greater than or equal to 0, Type Y construction enterprises will maintain their existing strategy. When the payoff difference is less than 0, it will change its strategy with a certain probability [30]. The probability Φ(*U*_*Y*_^*D*^ −  *U*_*N*_^*D*^) of changing the strategy is shown in the following formula:
  (1) $$\begin{array}{c} \Phi \left(U_{Y}^{D}-\;U_{N}^{D}\right)=\left\{\begin{array}{cc} \frac{\left(U_{Y}^{D}-\;U_{N}^{D}\right)}{U_{Y}^{D}}, & U_{Y}^{D}<U_{N}^{D},\\ 0, & U_{Y}^{D}\geq U_{N}^{D}. \end{array}\right. \end{array}$$
 Hypothesis 4: the expected average payoff of the construction enterprise that chooses the “*D*_Y_” strategy is *U*_*Y*_^*DA*^, and the expected average payoff of the construction enterprise that chooses the “*D*_N_” strategy is *U*_*N*_^*DA*^. Due to the different qualifications and capabilities of each construction enterprise, their real payoff will also be differentiated. Assume that the payoff of Type Y construction enterprise is *U*_*Y*_^*D*^= *λ*_*Y*_*∗U*_*Y*_^*DA*^, and the payoff of Type N construction enterprise is *U*_*N*_^*D*^=*λ*_*N*_*∗U*_*N*_^*DA*^. *λ*_*Y*_, *λ*_*N*_ are the influence coefficients of expected average payoff.
 Hypothesis 5: hypothesis *p* is the probability of the construction enterprise adopting PB mode. Using $\bar{x}$ to represent the derivative, the replication dynamic equation of the basic dynamic change rate at which the construction enterprise may choose to “*D*_*Y*_” the strategy can be expressed as

(2) $$\begin{array}{c} {\bar{x}}_{Y}=x_{Y}*x_{N}\left[\Phi \left(U_{Y}^{D}-U_{N}^{D}\right)-\Phi \left(U_{N}^{D}-U_{Y}^{D}\right)\right]p. \end{array}$$

### 2.2. System Dynamics Model Based on Evolutionary Game

#### 2.2.1. Main Modules and Equations

The system dynamics model based on evolutionary game is constructed by Vensim PLE. The model consists of three main modules: the construction enterprise decision-making module, the construction enterprise payoff module, and the consumer decision-making module. As shown in Figure 2, the construction enterprise decision-making module and the construction enterprise payoff module have an interactive relationship with each other, and the consumer decision-making module has an impact on the construction enterprise payoff module. Among them, the construction enterprise decision-making module is constructed according to the assumption rules and logical relations of the evolutionary game part.

*(1) The Construction Enterprise Decision-Making Module*. In this module, each construction enterprise has different qualifications and abilities and will change its own decisions according to the development of the industry, so the time of their “*D*_*Y*_” may be inconsistent. Each construction enterprise will go through a certain period of observation and then choose a strategy that suits itself. According to the plan of the Chinese government, the construction target of PB in the next stage is 2025. Therefore, the longest observation and consideration time of the construction enterprise is 5 years, and the average observation and consideration time is 1.5 years. Based on the above data, the dynamic change rate after *D*_*Y*_ (*R*_*T*_) is set.

This model will use the relevant data of PB development planning in Jiangsu Province, China. According to statistics from the National Bureau of Statistics of China, the number of real estate construction enterprises in Jiangsu Province in 2018 was 6,723, of which 39 were state-owned real estate construction enterprises [31]. Since PB mode has been implemented in China for a short time, the priority to adopt PB mode is mainly state-owned real estate construction enterprises. Therefore, suppose that the number of construction enterprises that initially adopted PB mode is 39. This module includes two level variables, namely, the construction enterprise adopting PB mode (*D*_*Y*_) and the construction enterprise not adopting PB mode (*D*_*N*_). One rate variable is the adoption rate of PB mode (*D*_*R*_) obtained according to the replication dynamic equation *R*_*B*_ of evolutionary game. The model is shown in Figure 3, and the meaning of the symbols is shown in Table 1.

The main equations of this module are as follows:

(3) $$\begin{array}{c} D_{R}=D_{T}*R_{T},\\ R_{T}=\text{Delay Fixed}\left(R_{B},\text{Random Normal}\left(0,5,1\text{.}5,0.1,0\right),R_{B}\right),\\ R_{B}=\bar{x_{Y}}=x_{Y}*x_{N}\left[\Phi \left(U_{Y}^{D}-U_{N}^{D}\right)-\Phi \left(U_{N}^{D}-U_{Y}^{D}\right)\right]p,\\ D_{Y}=0.039+\int D_{R},\\ D_{N}=6\text{.}684-\int D_{R},\\ p=\text{Random Normal}\left(0,1,\text{0.}4,0.3,0\right). \end{array}$$

*(2) The Construction Enterprise Payoff Module*. The construction enterprise payoff module mainly involves the payoff of the construction enterprise that selects the “*D*_*Y*_” strategy (*U*_*Y*_^*D*^) and the “*D*_*N*_” strategy (*U*_*N*_^*D*^). The payoff of the construction enterprise mainly includes construction payoff and government subsidies. Construction payoffs are realized through consumers' choice to purchase, and government subsidies are realized through government subsidies for construction projects that adopt PB mode. According to the current market conditions, government subsidies to construction enterprises are affected by factors such as subsidy factors, prefabrication ratio, and construction area of unit buildings. The model types of the payoff module of the construction enterprise that selects the “*D*_*Y*_” strategy (*U*_*Y*_^*D*^) and the “*D*_*N*_” strategy (*U*_*N*_^*D*^) are similar. Therefore, this module takes the module that the construction enterprise selects the “*D*_*Y*_” strategy (*U*_*Y*_^*D*^) as an example. The model is shown in Figure 4, and the meaning of the symbols is shown in Table 1.

The main equations of this module are as follows:

(4) $$\begin{array}{c} U_{Y}^{DA}=\frac{\left[\left(P_{1}-C_{1}\right)*A_{R}*C_{1}^{C}\right]}{D_{Y}}+S,\\ S=\left\{\begin{array}{cc} A_{C}*s*f*100, & Z\geq 0.5,\;A_{C}*s*f*100\leq 1800,\\ 1800\text{,} & Z\geq 0.5,\;A_{C}*s*f*100>1800, \end{array}\right.\\ f=\left\{\begin{array}{cc} \left(D_{Y}-\text{Delay}1\left(D_{Y},\text{Time Step}\right)\right), & \left(D_{Y}-\text{Delay}1\left(D_{Y},\text{Time Step}\right)\right)\geq 0,\\ 0, & \left(D_{Y}-\text{Delay}1\left(D_{Y},\text{Time Step}\right)\right)<0. \end{array}\right.\\ U_{Y}^{D}=U_{Y}^{DA}*\lambda_{Y},\\ \lambda_{Y}=\text{Random Normal}\left(\text{0.}9\text{, }1\text{.}3\text{ , }1\text{, 0.}2\text{ , 0}\right). \end{array}$$

*(3) The Consumer Decision-Making Module*. The consumer decision-making module mainly characterizes the consumer's purchase decision for TB or PB, and its purchase decision mainly considers the price, construction quality, and delivery waiting time of construction products. Assuming that there are N types of developed construction products on the market, consumers will give priority to the construction products that can generate the greatest purchase motivation [32]. The consumer's purchase motivation function can be expressed by the following formula:

(5) $$\begin{array}{c} M_{i}=P_{i}*PS_{i}+Q_{i}*QS_{i}+W_{i}*WS_{i}+l_{i}. \end{array}$$

The price sensitivity distribution model shows that the lower the price of a product is, the less price sensitivity the product produces, that is, the smaller the obstacle to consumers' purchasing motivation [33]. The consumer's price sensitivity is an exponential function of the difference between the actual product price *P*_*i*_ and the expected price *P*_*e*_. Due to the different socioeconomic attributes *k* of different consumers, their expected price *P*_*e*_ is different. Therefore, the formula is as follows:

(6) $$\begin{array}{c} PS_{i}=-\alpha^{P_{i}-\left(P_{e}+k\right)},\\ k=\text{Random Uniform}\left(-0.2,0.1,0\right). \end{array}$$

The quality sensitivity distribution model is used to measure the extent to which the quality of TB products and PB products affect consumers' motivation to purchase the products [34]. According to Taguchi quality theory and related research [35], consumers' perception of construction product quality mainly involves two aspects, including construction management level and information technology level. Therefore, comprehensive consumers' perception of different quality factors will get consumers' overall quality evaluation of construction products. The overall quality evaluation formulas of different building modes are expressed as follows:

(7) $$\begin{array}{c} \mu_{i}=aQ_{i}^{2}+bQ_{i}+d,\\ Q_{i}=m_{i}t_{i},\\ QS_{i}=\beta^{\left|Q_{i}-Q_{e}\right|}. \end{array}$$

The delivery waiting time sensitivity distribution model is used to measure the extent to which the delivery time of different building modes affects consumers' motivation to purchase the product. *WS*_*i*_ is an exponential function of the difference between the actual delivery waiting time *W*_*i*_ and the expected delivery waiting time *W*_*e*_ of the building. Due to the different socioeconomic attributes *w* of different consumers, the expected delivery waiting time *W*_*e*_ is different. Therefore, the formula is as follows:

(8) $$\begin{array}{c} WS_{i}=\eta^{W_{i}-\left(W_{e}+w\right)},\\ w=\text{Random Uniform}\left(-0.5,0.5,0\right). \end{array}$$

The conditions for consumers to choose PB based on purchasing motivation are

(9) $$\begin{array}{c} C_{1}^{CC}=\left\{\begin{array}{cc} 1, & M_{1}\geq M_{2},\\ 0, & M_{1}<M_{2}. \end{array}\right. \end{array}$$

Under this condition, the number of consumers purchasing PB is

(10) $$\begin{array}{c} C_{1}^{C}=50+\int C_{1}^{CC}. \end{array}$$

The conditions for consumers to choose TB are

(11) $$\begin{array}{c} C_{2}^{CC}=\left\{\begin{array}{cc} 1, & M_{1}\geq M_{2},\\ 0, & M_{1}<M_{2}. \end{array}\right. \end{array}$$

The number of consumers purchasing TB is

(12) $$\begin{array}{c} C_{2}^{C}=100+\int C_{2}^{CC}. \end{array}$$

The model is shown in Figure 5, and the meaning of the symbols is shown in Table 1.

#### 2.2.2. System Dynamics Model

Based on the above three modules, the system dynamics model of PB mode adopted by Chinese construction enterprises is established. As shown in Figure 6, this model includes 4 level variables, 3 rate variables, 33 auxiliary variables, and 21 constants.

## 3. Model Simulation

### 3.1. Initial Value Setting and Simulation

This paper sets the initial value based on the current data of PB in Jiangsu Province, China. According to the “Thirteenth Five-Year Development Plan for the Modernization of Construction Industry in Jiangsu Province,” PB construction can apply for affordable housing projects, and for affordable housing projects built with PB, you can apply for a reward of no more than 300 yuan/m^2^. When the prefabrication ratio of reinforced concrete structures is not less than 40%, the project will be subsidized, and the maximum subsidy for a single project will not exceed 18 million yuan per unit. Since China has determined that the minimum prefabrication ratio of PB is 50%, this paper sets the minimum prefabrication ratio as 50%. The prefabrication ratio set in the model has a linear relationship with the construction cost, in which the linear scale coefficient is 0.56 [36]. Based on the literature [37], when the prefabrication ratio of PB is greater than or equal to 50%, the cost of each additional 1% increase in the prefabrication ratio is about 29 yuan. This paper assumes that the construction area of the initial new construction project is 30000 m^2^. According to the data query of China National Bureau of statistics in 2018, the average sales price of residential commercial housing is 10773.5 yuan/m^2^. This paper uses Vensim PLE software to set TIME STEP to 0.0078125, and the initial value setting is shown in Table 2.

According to the setting of the initial value, the result of the adoption of PB mode in the construction enterprise is shown in Figure 7. The simulation results show that the adoption of PB mode by construction enterprises will reach a peak of 3.566 in the fourth year, that is, 3566 construction enterprises will adopt PB mode in engineering projects. However, after reaching the peak, the construction enterprises that adopted PB mode fluctuated in the form of shocks and eventually decreased gradually at a lower rate.

### 3.2. Analysis of Different Influencing Factors

#### 3.2.1. Influencing Factors at the Government Level

*(1) The Impact of Government Subsidies*. In this experiment, we changed the value of the *D*_Y_ subsidy factor and set the value to 0, 0.01, and 0.02, respectively, that is, the subsidy of 0, 100, and 200 yuan per square meter for the PB project. The simulation results are shown in Figure 8. The higher the amount of subsidy, the higher the peak value of *D*_Y_ and the faster the growth rate.

The simulation results show that government subsidies play a relatively important role in promoting the maturity of PB market, but for an already mature stable market, the role of government subsidies is relatively small.

*(2) The Impact of the Publicity and Guidance of Government Policies*. In this experiment, we will analyze the impact of government policy propaganda and guidance on the adoption of PB mode by construction enterprises. We set the value of *g* to 0.1, 0.2, and 0.3, respectively, that is, the government has promoted consumers' favorability of PB mode by 10%, 20%, and 30% through publicity and guidance. The simulation results are shown in Figure 9. The government's publicity and guidance strength can play a positive role in promoting the results of the previous PB adoption, and the effects of different publicity and guidance strengths are not very different. However, in the later stages of the market, different publicity and guidance efforts will show differentiated promotion effects. The greater the strength is, the better the market will adopt PB.

Therefore, in the early stage of PB being introduced into the market, the government should adopt the way of subsidy to increase the market share of PB, while in the later stage of the market, the government should adopt the way of publicity and guidance to further promote the development of PB mode.

#### 3.2.2. Influencing Factors at the Construction Enterprise Level

*(1) The Impact of the Initial “D_Y_” Probability of the Construction Enterprise*. In this experiment, firstly, we set the probability of initial adoption of PB by the construction enterprise to 20%, 30%, 40%, and 50%, respectively. The simulation result is shown in Figure 10. At the initial stage of the formation of PB market, it is very important to improve the probability of the construction enterprise's initial adoption of PB mode to quickly improve the market share of PB, and the higher the initial adoption probability, the greater the peak value and fluctuation of the market share. However, the market share of PB will gradually reach a balanced and stable state. The probability that the construction enterprise initially adopts PB mode has no differential impact on the later market equilibrium. Therefore, the probability that the construction enterprise initially adopts PB mode does not have a first-mover advantage for the final market share of PB mode.

*(2) The Impact of the Information Technology Level*. In the scenario where *m*_1_ in the quality factor is set to 1, we set the value of *t*_1_ in the quality factor to 1, 1.5, and 2, respectively, which means that the information technology level in the PB product quality factor is increased by 0%, 50%, and 100%, respectively. The simulation result is shown in Figure 11.

The results show that in the early process of the adoption of PB mode, different information technology levels have little impact on the market share of PB. However, in the later stages of the market, different information technology levels have had a different effect on the adoption of PB. When *t*_1_ increases from 0% to 50%, the growth rate of PB market share is greater than that when *t*_1_ increases from 50% to 100%. It can be seen that the construction enterprise should follow the principle of moderation when deciding on the information technology level, and that too high information technology level has a limited effect on advancing the PB market share.

*(3) The Impact of Quality Factors*. In this part, we will analyze the comprehensive influence of construction management level and information technology level on the adoption of PB mode. First, we set the value of *m*_1_ to 1.5 (the initial value of *m*_1_ is 1). On this basis, we set the value of *t*_1_ to 1, 1.5, and 2, respectively. The simulation result is shown in Figure 12.

As can be seen from the figure, the market share of PB mode shows a rapid rise and then a decline and a slow rise. Compared with Figure 10, when the value of *m*_1_ is set to 1.5, the overall *D*_*Y*_ number is further improved. In the scenario where the value of *m*_1_ increases, a higher *t*_1_ will bring a larger PB market share. When *t*_1_ increases from 0% to 50%, the increase in PB market share is greater than the increase when *t*_1_ increases from 50% to 100%. It can be seen that increasing *m*_1_ and *t*_1_ will play a superimposed role in promoting the growth of PB market share.

*(4) The Impact of Price Factors*. In this experiment, we change the value of *P*_1_ to *P*_1_−0.1 and *P*_1_+0.1, that is, the price of PB products per square meter is reduced by 1,000 yuan or increased by 1,000 yuan. The simulation results are shown in Figure 13, and the market share of PB mode shows an evolutionary trend of rapid rise and then slow decline.

Reducing the value of P_1_ can quickly increase the market share of PB in a short period of time and enable it to reach a higher share. However, after reaching the peak, the market share of PB has shown a slow downward trend. It can be seen that adopting a low-price strategy will help PB mode to quickly penetrate the market, but for the later stage of the market, the ability of price to further enhance the market share of PB is limited.

*(5) The Impact of Delivery Waiting Time Factors*. We set the value of *W*_1_ to 0.75, 1, and 1.25, respectively, that is, the delivery waiting time of PB is set to 0.75, 1, and 1.25 years. The simulation result is shown in Figure 14. It can be seen from the figure that under the condition that consumers set in this paper have the same sensitivity to product price, quality, and delivery waiting time, different delivery waiting times have little difference on the market share of PB. However, in the early stage of the market, the delivery waiting time has a certain impact on the peak of the PB market share, but this differential impact is not very obvious.

## 4. Discussion

In the above simulation results and analysis, it can be found that the changes of different factors will have a different impact on the adoption strategy of the construction enterprise. It is necessary to analyze the most favorable aspects of different factors affecting the construction enterprise's adoption of PB mode from different angles. This paper will analyze the influencing factors from the following perspectives.

### 4.1. Influencing Factors at the Government Level

From the perspective of changing government subsidies, government subsidies play a positive role in promoting construction enterprises to adopt PB mode, especially in the initial stage of adopting PB mode by construction enterprises, which confirms Li et al.'s research results [14]. Also, the higher the government subsidy is, the higher the peak value of construction enterprises adopting PB mode is and the longer it will continue to grow. However, for the PB market that has gradually stabilized, government subsidies have no obvious promoting effect. Timely reduction or termination of government subsidies can effectively reduce fiscal expenditures and achieve good market effects.

From the perspective of improving the publicity and guidance of government policies, the government's positive guidance for PB mode has improved consumers' favorability of PB mode, which in turn promoted the long-term and steady development of the PB market, which is consistent with Wang et al.'s research results [26]. This effect is not obvious in the initial stage of the PB market but gradually widened the gap in the later stage. Positive publicity and guidance have a subtle effect on the development of the PB market, and the longer the time, the more obvious the effect.

In summary, in the early stage of PB mode entering the market, the government should use subsidies to increase the market share of PB. Although the publicity and guidance of government policies are more obvious in the later stage of the PB market, the government should still adopt positive publicity and guidance methods in the early stage of the PB market to further promote the development of PB mode.

### 4.2. Influencing Factors at the Construction Enterprise Level

From the perspective of changing the initial acceptance probability of the construction enterprise, higher initial acceptance probability of the construction enterprise is of great significance to the formation of the initial PB market, which is conducive to the rapid improvement of the maturity of the PB market. However, excessive pursuit of the probability of construction enterprises initially adopting PB mode is not conducive to the stable development of the PB market. In the long run, the adoption intention of the construction enterprise should follow a step-by-step process and maintain a relatively stable growth trend.

From the perspective of changing the level of information technology, the improvement of the level of PB construction information technology has significantly accelerated the rate at which construction enterprises adopt PB mode. However, the degree of improvement in the level of PB construction information technology is not linearly related to the rate at which construction enterprises adopt PB mode. When the PB construction information technology level is raised to a higher level, the impact of the increase in the PB construction information technology level on the increase in the rate of the construction enterprise adopting PB mode will show a decreasing trend under the same proportion each time. Therefore, it is necessary to uphold the principle of moderation for the improvement of the information technology level, and blindly pursuing the unilateral improvement of the information technology level may not achieve the expected results.

From the perspective of changing quality factors, when the level of PB construction management improves, the corresponding improvement in the level of construction information technology will have a significant impact on accelerating the increase in the rate at which construction enterprises adopt PB mode. While maintaining the improvement of the construction management level, the improvement of the same proportion of the information technology level will sharply reduce the increase in the rate of construction enterprises adopting PB mode. It can be seen that the improvement of the construction management level has a positive effect on the adoption of PB mode by the construction enterprise, and the improvement of the construction management level and the information technology level at the same time will facilitate the rapid development of PB mode and maintain the PB market share for a long time.

From the perspective of changing price factors, compared with increasing the price of PB per square meter, the price reduction has shown an advantage in the early stage of the PB market. The price lower than the market price has been supported by more consumers, which has affected the construction enterprise's adoption of PB mode. Therefore, the price factor has a more direct impact on the PB market, and the lower price indirectly stimulates the construction enterprises to improve the adoption of PB mode.

From the perspective of changing the delivery waiting time factor, the reduction in PB delivery waiting time does not significantly affect the rate at which construction enterprises adopt PB mode. This also shows to a certain extent that when the delivery waiting time of the building is within the consumer's tolerance range, it will not cause strong rejection due to the long delivery waiting time. Therefore, the impact of the delivery waiting time factor on the construction enterprise's adoption of PB mode is not significant.

To sum up, we can draw the following conclusions. Firstly, the initial adoption intention of the construction enterprise should adopt the strategy of gradual improvement. Secondly, the construction management level and the information technology level in the quality factor of PB have complementary effects. At the same time, their improvement can not only quickly increase the PB market share but also maintain the stable and good development of the PB industry. Thirdly, the reduction of the price factor is conducive to the rapid increase of the PB market share in the short term. Fourthly, the delivery waiting time factor will not have a major impact on the construction enterprise's adoption of PB mode.

## 5. Conclusions and Recommendations

PB has developed earlier in some developed countries, such as the United Kingdom and the United States, and already has a certain market scale [38]. However, PB mode is still in the ascendant in China, but based on the needs of China's energy saving, emission reduction, and green development, PB mode has attracted the attention of many scholars in recent years.

Combined with evolutionary game theory, this study establishes a system dynamics model of Chinese construction enterprises' adoption behavior of PB mode under the scenario of multiagent interaction and uses the data of Jiangsu Province in China for simulation analysis. The purpose is to clarify the behavior mechanism of Chinese construction enterprises' adoption of PB mode and the evolution law of PB market share, so as to provide a certain theoretical basis for the vigorous development of PB mode in China. The corresponding conclusions and recommendations are as follows:

1. Government subsidies play an important role in promoting the maturity of the PB market. Maintaining certain government subsidies can ensure a longer and more stable market share of PB mode. However, for the already more mature market, the role of government subsidies is relatively small. Therefore, government subsidies can be gradually reduced or cancelled after promoting the development of PB mode to achieve a good market effect. At the same time, the publicity and guidance of government policies have gradually produced the effect of promoting the market share of PB, which requires the accumulation of preliminary work. Therefore, in the early stage of the introduction of PB mode to the market, the government should simultaneously provide subsidies to construction enterprises and publicize and guide consumers to increase the market share of PB and further promote the development of PB mode.
2. The initial acceptance probability of the construction enterprise should not be excessively pursued. The higher the initial probability of adoption, the greater the peak of the PB market share and the greater the volatility, which is not conducive to the stable development of the PB industry. Also, the probability that the construction enterprise initially adopts PB mode has no differential impact on the later market equilibrium state. Different initial acceptance probabilities of the construction enterprise will make the market share of PB reach a gradually balanced and stable state. Therefore, the probability that the construction enterprise initially adopts PB mode does not have a first-mover advantage for the final market share of PB mode.
3. The reduction of the price factor can quickly increase the market share of PB mode in a relatively short period of time. However, in the later stages of the market, lowering the price factor has limited ability to further increase PB's market share. The reduction of price factors cannot maintain the lasting and stable development of the PB market. The simultaneous improvement of the construction management level and the information technology level in the quality factors has an important impact on the market share of the later stage of PB mode and can maintain the steady growth of the PB market. Compared with price factors and quality factors, the delivery waiting time factor has no significant impact on the market share of PB mode. Therefore, the delivery waiting time factor does not need to be considered more by the construction enterprise in the decision to adopt PB mode. In summary, the PB industry still needs to promote the development of PB with the promotion of quality improvement as the main direction. Under the premise of small price fluctuations and stable quality improvement, the reduction in delivery waiting time should be gradually reduced, so that the PB industry can go more stable and go further.

This paper also has some limitations. For example, the model does not consider the specific components of construction cost, the relationship and behavior of other stakeholders, etc. In addition, this paper mainly studies the adoption behavior of PB mode by Chinese construction enterprises and comes to the conclusion that the universality and reference significance of management conclusions need to be strengthened. In the future, we can consider the relationships and behaviors between more stakeholders, add more abundant influencing factors, and promote the steady development of PB.

## Figures and Tables

**Figure 1:** System analysis of construction mode selection of construction enterprise.

**Figure 2:** Interaction between modules.

**Figure 3:** System diagram of the decision-making module of the construction enterprise.

**Figure 4:** System diagram of the payoff module of the construction enterprise.

**Figure 5:** System diagram of consumer decision-making module.

**Figure 6:** The system dynamics model of adoption behavior of PB mode by Chinese construction enterprises.

**Figure 7:** Initial simulation results.

**Figure 8:** Simulation results of changes in government subsidies.

**Figure 9:** Simulation results of changes in government policy publicity and guidance.

**Figure 10:** The simulation result of the initial “*D*_Y_” probability change.

**Figure 11:** Simulation results of changes in the information technology level.

**Figure 12:** Simulation results of quality factors.

**Figure 13:** Simulation results of changes in price factors.

**Figure 14:** The simulation result of the change of the delivery waiting time factor.

**Table 1:** The symbolic meaning of the main equations.

Symbol	Implication
*D*_*R*_	PB application rate
*D*_*T*_	Total number of construction enterprises
*R*_*T*_	Dynamic change rate after *D*_*Y*_
*R*_*B*_	Basic dynamic change rate of *D*_*Y*_
*p*	Initial probability of *D*_*Y*_
*U*_*Y*_^*DA*^	Average expected payoff of *D*_*Y*_
*C*_*i*_	Cost for per square meter of *i*(*i*=1 is PB; *i*=2 is TB)
*P*_*i*_	Price for per square meter of *i*
*S*	Subsidies for *D*_*Y*_
*A*_*R*_	Average building area of per suite
*A*_*C*_	Building area of unit building
*C*_*i*_^*C*^	Consumers of choosing *i*
*Z*	Prefabrication ratio
*U*_*Y*_^*D*^	Expected payoff of *D*_*Y*_
*s*	Subsidy per square meter of *D*_*Y*_
*f*	The amount of change of per unit time of *D*_*Y*_
*M*_*i*_	Consumers' motivation to purchase *i*
*PS*_*i*_	Consumers' price sensitivity parameters for *i*
*Q*_*i*_	Quality of *i*
*QS*_*i*_	Consumers' quality sensitivity parameters for *i*
*W*_*i*_	Delivery waiting time for *i*
*WS*_*i*_	Consumers' delivery waiting time sensitivity parameters for *i*
*l*_*i*_	The degree of external influence of consumers purchasing *i*
*P*_*e*_	Consumer expected price for per square meter of building
*k*	Consumers' socio-economic attributes of price factors
*μ*_*i*_	The quality to cost ratio of *i*
*m*_*i*_	Management level in *i* construction
*t*_*i*_	Information technology level in *i* construction
*Q*_*e*_	Consumer expected quality for building
*a*, *b*, *d*	Constant
*W*_*e*_	Expected delivery wait time for consumers
*w*	Consumers' socio-economic attributes of delivery waiting time factors
*C*_*i*_^*CC*^	Probability of consumers choosing *i*

**Table 2:** Setting of initial simulation value.

Variable	Category	Initial value	Unit
Initial value of *D*_*Y*_	Level	0.039	Thousand
Initial value of *D*_*N*_	Level	6.684	Thousand
*D*_*T*_	Constant	6.723	Thousand
*λ*_*Y*_	Constant	1	1
*λ*_*N*_	Constant	1	1
*P*_1_	Constant	1.07735	Ten thousand yuan
*P*_2_	Constant	1.07735	Ten thousand yuan
*P*_*e*_	Constant	0.8	Ten thousand yuan
*W*_1_	Constant	1.5	year
*W*_2_	Constant	2	year
*W*_*e*_	Constant	1	year
*t*_1_	Constant	1	1
*t*_2_	Constant	1	1
*m*_1_	Constant	1	1
*m*_2_	Constant	1	1
*Q*_*e*_	Constant	3	1
*A*_*C*_	Constant	30000	m^2^
*A*_*R*_	Constant	100	m^2^
*Z*	Constant	0.5	1
*s*	Constant	0.03	Ten thousand yuan
*g*	Constant	0	1

## Data Availability

The data used to support the findings of this study are available from the corresponding author upon request.
